This article has been retracted.

# Exploring the transactive relationships of influence factors for online asynchronous learning transactive memory system

**DOI:** 10.1016/j.heliyon.2024.e36441

**Published:** 2024-08-21

**Authors:** Jiao Zhang, Min Zhao, Liang Wang

**Affiliations:** a School of Foreign Languages, Dalian Polytechnic University, Dalian, 116034, China; b School of Maritime Economics and Management, Dalian Maritime University, Dalian, 116026, China

**Keywords:** Online asynchronous learning, Transactive memory system, Influence factors, Transactive relationships, Structural equation modeling

## Abstract

Transactive memory system (TMS) makes learning and transferring knowledge easy and efficient. This study has constructed a conceptual model of TMS to reveal the crucial factors influencing the formation of a TMS in online asynchronous learning to foster knowledge sharing and collaboration and enhance knowledge transfer effectiveness. The conceptual model of TMS is built upon theoretical foundations concerning the creation of TMS and the variables influencing them. The study has put forth a set of hypotheses to predict the expected effects of group factors, individual factors, task interdependence, the degree of intellectual silence, and knowledge management on the formation of TMS. In this study, a total of 229 questionnaire data were collected from undergraduate, master's, and doctoral students in Northeast China who had experience with an online asynchronous learning TMS. Structural equation modeling has been employed to identify the key indicators involved and their influence on the formation of TMS. The empirical study was carried out using statistical analysis of SPSS data, with the results indicating that each factor has varying impacts on knowledge management, ultimately affecting the formation of TMS. These findings provide a more nuanced understanding of how these factors shape online asynchronous learning environments.

## 1 Introduction

In the post-epidemic era of information explosion and knowledge transference, learning is no longer confined to traditional classrooms or training courses. A new wave of educational revolution and rapid transformation of learning modes is underway, driven by the continuous advancement of innovative technologies such as artificial intelligence, Internet technology, big data, and 5G [1]. Online asynchronous learning has ushered in a paradigm shift in teaching and learning, enhancing the integration and transfer of knowledge across temporal and spatial divides between educators and students [2]. The best practices of active, blended, and collaborative learning have been seamlessly integrated into online asynchronous learning platforms to facilitate students' acquisition of conceptual knowledge and enhance their problem-solving skills [3]. This, in turn, empowers learners to attain higher-order cognition for knowledge sharing [4]. Efficient knowledge transfer within asynchronous learning environments plays a pivotal role in improving the effectiveness of teaching and learning and enhancing memorization. Developing the ability to interact with knowledge asynchronously accelerates learners' knowledge retention, especially in scenarios with a spatial and temporal separation between the teacher's instruction and the student's learning [5].

Transactive memory system (TMS), which involves the division of labor and collaboration based on individuals' perceptions [6] of each other's knowledge mastery, significantly impacts learners' knowledge acquisition and fosters innovative cooperation [7]. As a knowledge-sharing system that enhances the memory retention of online learners and addresses issues of knowledge or information asymmetry among members, it involves the complementary transfer and efficient knowledge utilization within the student group. When members require knowledge in a specific area, they can readily connect with others with expertise in that domain, seeking assistance or information [8]. Therefore, the study of online asynchronous learning TMS helps to enhance the personalized learning experience and memory effect promotes the innovation of education mode, and is of great significance in improving learners' motivation and learning effectiveness.

Researchers continually strive to enhance online asynchronous learning TMS in response to the increasing demand for online education. This is achieved by amalgamating personalized learning [9], principles derived from cognitive science, transactive communities, and real-time feedback to create a more effective and productive learning experience [[10], [11], [12]]. These measures aim to assist learners in mastering knowledge and skills. While existing research explores aspects related to the online asynchronous learning TMS's concepts and components of conceptual model construction [13], which lacks a comprehensive theoretical framework. This study systematically analyzes the conceptual model of interactive memory for online asynchronous learning. It develops a theoretical framework that fills the gaps in current incomplete theoretical frameworks and research on flexibility, personalized learning [14,15], and the application of cognitive science [16] to traditional educational models [17].

Additionally, scholars have also devoted attention to the various influencing factors among user members of TMS [18]. However, there is a limited exploration of the transactive relationships between these factors. Consequently, further research is needed to identify and categorize these influencing factors and systematically analyze their intrinsic logical relationships.

Hence, in order to reveal the formation mechanism of learners' TMS and promote the transformation of the educational model, this study will comprehensively explore the generation mechanism and influencing factors of online asynchronous learning TMS, addressing the following two research questions.

(1) What is the formation process of online asynchronous TMS?
(2) What are the key factors influencing the formation of online asynchronous TMS?

To address the above questions, this study analyzes the concepts, influencing factors, and formation process of interactive memory systems to promote personalized learning and innovation in educational models.

The upcoming structure of this study is as follows: Section 2 will analyze previous research on online asynchronous learning TMS. Section 3 will construct a theoretical TMS model, including identifying influencing factors, and develop a path model based on the proposed research hypotheses. Section 4 will empirically assess the model's fit and validate the accuracy of the research hypotheses. Section 5 will explore the implications of the research findings. Finally, Section 6 will present the conclusions.

## 2 Previous research on online asynchronous learning TMS

### 2.1 Conceptual model of online asynchronous learning TMS

Online asynchronous learning involves separating teacher-led activities and student-led learning across spatial and temporal dimensions, serving as a crucial mode of collaborative learning [19]. Within this context, the TMS is a concept rooted in external memory. Wegner has been pioneering in exploring TMS since 1985 and was the first scholar to undertake extensive research on and provide definitions for TMS. The TMS can be likened to a knowledge network [20]. This network's formation stems from the diverse professional knowledge that online learning participants employ to exchange data, information, and knowledge amongst one another, ultimately leading to the integration and utilization of knowledge. Concurrently, the TMS is a platform for learners, enabling them to store and retrieve information [21].

The TMS comprises three fundamental dimensions: expertise, trustworthiness, and coordination. Achieving an efficient TMS necessitates the balanced and consistent advancement of these three dimensions. The harmonious progression of expertise, trustworthiness, and coordination is paramount to ensuring the system's effectiveness [22]. This complementary development of the three dimensions forms the cornerstone of the process involved in constructing the conceptual model of transactive memory.

While the conceptual model provides us with an abstract understanding of the operational mechanisms of the TMS, exploring the critical influences of the TMS is the embodiment of the abstraction of the concrete.

### 2.2 Influences of TMS

Both domestic and international scholars have conducted comprehensive and in-depth research on the factors that influence TMS. Orr's [23] work underscores the pivotal role of communication in facilitating the exchange of knowledge, lessons, and experiences among learning members. He posits that continuous and effective communication among these members fosters the development of shared memories, which, in turn, underpin the exchange of knowledge and lessons, as well as cooperative efforts based on these shared memories.

Within the context of online asynchronous learning, it has been argued that active and effective communication among learning members significantly contributes to the formation of TMS [24]. Furthermore, some scholars [13] contend that there exists a web of interdependence among learning members, with the learning and memory processes of these members intersecting and mutually influencing one another. Zhang et al. [25] sampled 104 learning teams across various fields and demonstrated a positive correlation between task interdependence, the interdependence of cooperative goals, and support for innovation with the team's TMS.

### 2.3 Formation of TMS

TMS's theoretical foundations and influencing factors are examined, facilitating a more in-depth exploration of its formation process. Regarding the formation process of TMS, Chinese and international scholars generally share consistent perspectives. Wegner, an early and in-depth researcher in this field, posits that the TMS effectively enhances learners' knowledge retention, reduces redundancy, and improves memory effectiveness through the coordination and collaboration of learning members. He also outlines that the formation of TMS primarily involves three stages: the directory updating stage, the knowledge distribution stage, and the retrieving coordination stage. This framework has garnered widespread recognition and application by subsequent scholars studying TMS. For instance, Gupta [26] investigated the connections and mechanisms of these three formation phases, thereby enriching the relevant theories on TMS formation.

Traditional learning styles influence most adult learners and tend to learn by observing others' transactions. The interest and proficiency of core participants primarily determine the direction and depth of these transactions. The contribution of social transactions to effective learning is still an area that requires improvement [27]. Developing knowledge-sharing and memory-transactive systems among students in online asynchronous environments warrants further exploration and research.

## 3 Model construction of online asynchronous learning TMS

### 3.1 Conceptual model

Wegner [28] introduced the connotation of transactive memory in the 1980s to elucidate the behaviors of close friends, colleagues, and couples who exchange valuable information. Some studies indicate that the TMS is a collective system for encoding, storing, and retrieving coordination [29]. Its formation consists of the following three stages: directory updating (Specialization. Understanding who among the team members possesses what knowledge i.e., knowledge differentiation or memory specialization), knowledge distribution (Credibility. Assigning new information to those among the team members who are best suited to store it, this reflects task credibility, with members trusting each other's knowledge and expertise), and retrieving coordination (Coordination. How to find expertise knowledge and integrate and utilize it, emphasizing coordination, members know who knows what and does what for the team to work together smoothly and efficiently. The third dimension of TMS is coordination).

Argote et al. [30] state that the directory updating, knowledge distribution, and retrieving coordination within the TMS align with the stages of encoding, storing, and retrieving information, respectively. In the encoding stage, learning members continually update their cognitive directory by encoding knowledge and the individuals with whom they share that knowledge. This process is akin to building cognitive maps. During the storing stage, the emphasis lies on organizing newly acquired knowledge for storage alongside relevant peers, facilitating the most suitable distribution of knowledge. In the retrieving information stage, learning members must engage in solidarity and collaboration to retrieve the necessary information from other members. These three phases (encoding, storing, and retrieving information) are carried out cyclically to ensure the efficient functioning of the TMS. The resulting conceptual model of the TMS is illustrated in Fig. 1.

**Fig. 1:** Conceptual model of online asynchronous learning TMS

### 3.2 Hypothetical model construction

#### 3.2.1 Formulation of the research hypothesis

(1) Hypotheses on task interdependence, knowledge management, and degree of intellectual silence about the effectiveness of the interactive memory system

**Task interdependence**: Gupta [26] argues that task interdependence is a crucial factor in knowledge creation and storage, it positively affects the transmission and transfer of knowledge in TMS. The intertwining of knowledge from different domains is instrumental in facilitating knowledge creation, as it opens the potential for cross-domain inspirations, where discoveries in one area can trigger fresh ideas in another [31]. In teams with high task interdependence, members frequently exchange information and coordinate their work, improving the efficiency of information sharing and the quality of communication. Therefore, the effectiveness of the interactive memory system will be more demanding in situations with a high degree of task interdependence.

**Knowledge management**: It includes the knowledge creation, knowledge storage, and knowledge transfer, TMS can be continually expanded and updated when team members can continually generate new knowledge (encoding), knowledge storage enables knowledge to be efficiently recorded and managed (storing), and transferring knowledge helps team members to share and transfer knowledge (retrieving information). Thus, knowledge management positively affects TMS.

**Intellectual silence**: The degree of intellectual silence can constrain knowledge creation and transfer. When knowledge is challenging to comprehend and absorb by in-group learners, it disrupts the natural flow of knowledge within the learning community, thus impeding the formation of a transactive memory and causing negative effects. Thus, a high level of intellectual silence that makes knowledge difficult to understand by the group will hinder the formation of the effectiveness of the TMS and have a negative impact.

(2) Hypotheses related to the effectiveness of group factors and TMS

Group factors are pivotal in shaping the dynamics of the TMS.

**Group learning**: Firstly, group learning is a process that induces changes in the knowledge levels of its members and the interactions and communications between them [32]. This, in turn, fosters communication among members, enhancing mutual understanding and mutual support [33]. It facilitates the creation and transfer of new knowledge, which serves as the bedrock for the TMS.

**Group communication**: It serves as a crucial mechanism for fostering the formation of the TMS. Carlynn et al. [34] contend that positive and effective communication is fundamental to successful collaboration. Through open and efficient communication, members can exchange insights, perspectives, and experiences. This information exchange perpetuates the continuous creation and transfer of knowledge within the group, elevating the quality and utility of the TMS.

**Membership trust**: It is another pivotal factor in the formation of the TMS. Rousseau et al. [35] posit that trust is a willingness to accept the information provided by others and is a psychological process grounded in cognitive, motivational, and affective factors [36]. The transfer of knowledge between group members relies on this trust, and enhancing trust levels among members facilitates the flow and assimilation of knowledge within the group.

**Group cohesion**: It contributes to the stability and longevity of the TMS. Man argues that strong group cohesion enhances team awareness and fosters knowledge creation and transfer among members [37]. It ensures the TMS's long-term existence and ongoing development.

(3) Hypotheses related to individual factors to the effectiveness of TMS

Individual factors, specifically knowledge stock and shared willingness, hold a critical role in knowledge creation and transfer and are among the core drivers in the formation of TMS.

**Knowledge stock**: Knowledge stock represents the wealth of knowledge and experience accumulated by individuals or organizations over time. These stocks provide valuable resources for innovation and problem-solving, serving as the foundation for generating new knowledge.

**Shared willingness**: The true value of knowledge lies in sharing and disseminating it to others, rather than hoarding it within individual minds or isolated groups. This culture of willingness to share fosters the flow and exchange of knowledge, ultimately spurring the creation and transfer of knowledge. The development of TMS hinges on more than just individual memory; it necessitates a collective reservoir of knowledge maintained by the entire learning community. Therefore, knowledge stock and shared willingness are not only vital for knowledge creation and transfer but also play a pivotal role in instigating and evolving TMS.

The above analysis framework is based on existing literature and facts, and research hypotheses are made as shown in Table 1.

**Table 1:** Impact factor role Assumptions.

Influencing factors	Hypothesis	Specific hypothetical elements
Task interdependence and the effectiveness of TMS	H1	Task interdependence is positively related to the effectiveness of TMS
Effectiveness of Knowledge Management and TMS	H2a	Knowledge creation is positively related to the effectiveness of TMS
	H2b	Knowledge storage is positively correlated with the effectiveness of TMS
	H2c	Knowledge transfer is positively correlated with the effectiveness of TMS
Intellectual silence and the effectiveness of TMS	H3	Intellectual reticence can hinder the effectiveness of TMS from increasing, with negative effects.
Group Factors, Knowledge Management, and the Effectiveness of TMS	H4a	Group learning promotes knowledge creation and ultimately positively affects the effectiveness of TMS
	H4b	Group learning promotes knowledge transfer and ultimately positively affects the effectiveness of TMS
	H4c	Group communication promotes knowledge creation and ultimately positively affects the effectiveness of TMS
	H4d	Group communication promotes knowledge transfer and ultimately positively affects the effectiveness of TMS
	H4e	Membership trust promotes knowledge storage and ultimately positively influences the effectiveness of TMS
	H4f	Membership trust promotes knowledge transfer and ultimately positively affects the effectiveness of TMS
	H4g	Group cohesion promotes knowledge storage and ultimately positively influences the effectiveness of TMS
	H4h	Group cohesion promotes knowledge transfer and ultimately positively affects the effectiveness of TMS
Individual Factors, Knowledge Management, and the Effectiveness of TMS	H5a	Knowledge stock promotes knowledge creation and ultimately has a positive impact on the effectiveness of TMS
	H5b	Shared willingness promotes knowledge transfer and ultimately positively affects the effectiveness of TMS

#### 3.2.2 Hypothetical model

The research hypotheses for each influencing factor are presented in Table 1. These hypotheses in the table serve as the foundation for constructing the online asynchronous learning TMS and forming the hypothesis model.

As shown in Fig. 2, the independent variables encompass group learning, group communication, membership trust, group cohesion in group factors, knowledge stock, shared willingness in individual factors, task interdependence, and intellectual silence. The mediating variables include knowledge creation, storage, and transfer within knowledge management. The dependent variable is the effectiveness of the TMS.

**Fig. 2:** Hypothetical model of online asynchronous learning TMS formation.

#### 3.2.3 Measurement of research variables

##### 3.2.3.1 Group factors

(1) Group learning

Drawing from the insights of Izci and Muslu [38], effective management of group learning involves analyzing and evaluating the impact of group learning. This entails considering the accumulation and expansion of individual and group knowledge, along with the enhancement of group learning capabilities and management. Building upon these principles, a Group Learning Measurement Scale was developed and is detailed in Table 2.

(2) Group communication

**Table 2:** Group learning measurement scale.

Variables	Label	Definition
Group learning	QT1	We will often have online group learning
	QT2	I learned what I needed to know through online group learning
	QT3	Through online group learning, the exchange of knowledge between me and other students has become much greater

Regular communication among peers within a group fosters knowledge creation and transfer, while also elevating the degree of comprehension and collaboration among learning participants. Learner-to-learner communication enhances individual knowledge-sharing and problem-solving within the learning context. Consequently, a corresponding measurement scale for group communication has been devised, and it is presented in Table 3.

(3) Membership trust

**Table 3:** Group communication measurement scale.

Variables	Label	Definition
group communication	GT1	I will take the initiative to consult with other classmates when I encounter learning problems that I don't understand.
	GT2	There are frequent discussions between our learning communities about a particular issue
	GT3	When problems arose, we were always able to work together as a group to solve them.

Trust forms the cornerstone of knowledge transfer among learning participants. As demonstrated in Shapiro's study [39], learners' comprehensive understanding of each other's knowledge and attributes hinges on mutual trust. This understanding has prompted the development of the Membership Trust Measurement Scale, which is illustrated in Table 4.

(4) Group cohesion

**Table 4:** Membership trust measurement scale.

Variables	Label	Definition
Membership trust	XR1	For information provided by other students in the study group, I think it is trustworthy
	XR2	I believe that the specialized knowledge and abilities of the students in the study group
	XR3	In group discussions, we rarely doubt the veracity of each other's information

Group cohesion is typically assessed using four key dimensions: the attractiveness of the group, the extent of mutual liking between individuals, the degree of individual pride in the group, and the level of individual loyalty to the team [40]. These dimensions have informed the creation of the Group Cohesion Measurement Scale, as presented in Table 5.

**Table 5:** Group cohesion measurement scale.

Variables	Label	Definition
Group cohesion	NJ1	I like online asynchronous learning for knowledge acquisition
	NJ2	I enjoy the knowledge transfer atmosphere of online asynchronous learning
	NJ3	I am willing to actively share my knowledge base to solve group learning tasks

##### 3.2.3.2 Individual factors

(1) Knowledge stock

An individual's existing knowledge reservoir plays a significant role in their capacity to assimilate new knowledge and enhance the overall knowledge level of the group. This, in turn, impacts the effectiveness of knowledge creation and transfer. Furthermore, an individual's knowledge stock also influences the extent of expertise variation within the TMS. Consequently, a Knowledge Stock Measurement Scale has been formulated, and it is detailed in Table 6.

(2) Shared Willingness

**Table 6:** Knowledge stock measurement scale.

Variables	Label	Definition
Knowledge stock	CB1	I have a certain amount of relevant knowledge base
	CB2	Members of our learning community have a reservoir of expertise in which they specialize
	CB3	The stock of knowledge possessed by different members of the group all play a role in the achievement of learning goals

A heightened willingness to share knowledge is highly advantageous for knowledge transfer, information dissemination, and promoting communication and mutual assistance among group learning members. It also facilitates a greater degree of coordination and cooperation within the TMS. Consequently, a Shared Willingness Scale has been developed, as detailed in Table 7.

**Table 7:** Shared willingness measurement scale.

Variables	Label	Definition
Shared willingness	GX1	When I encountered learning problems, I was eager to seek knowledge and help from other students
	GX2	I am willing to share my knowledge base with other students in the group study

##### 3.2.3.3 Task interdependence

A heightened level of task interdependence indicates that group learning participants rely extensively on one another, leading to increased knowledge dependence. This fosters collaborative cooperation among individuals and promotes the formation of TMS. Accordingly, the Task Interdependence Measurement Scale has been developed and is presented in Table 8.

**Table 8:** Task interdependence measurement scale.

Variables	Label	Definition
Task interdependence	HY1	Many learning tasks always require the cooperation of many learners to complete them
	HY2	I need the help and cooperation of other students to complete a learning task

##### 3.2.3.4 Knowledge management

(1) Knowledge creation

The four facets of "collectivization, internalization, integration, and externalization" concerning knowledge signify the process of knowledge creation within group learning. This process also reflects the continuous exchange, learning, and accumulation of knowledge by members of the learning community, contributing to the ongoing augmentation of expertise differences. Consequently, a Knowledge Creation Measurement Scale has been developed, and it is detailed in Table 9.

(2) Knowledge storage

**Table 9:** Knowledge creation measurement scale.

Variables	Label	Definition
knowledge creation	CZ1	My knowledge and skills have been enhanced by the communication and learning among the members of the group
	CZ2	Some of my knowledge comes from other students in the learning group
	CZ3	Teachers assign different kinds of new knowledge to different students for learning

The utilization of information technology or textbooks for knowledge storage, coupled with the creation of knowledge maps and expertise catalogs within the knowledge storage mechanism, facilitates the efficient retrieval of required knowledge or the identification of classmates knowledgeable in specific areas when students within the learning community have knowledge needs. Additionally, this system enables the timely updating of the knowledge directory. To measure these aspects, a Knowledge Storage Measurement Scale has been designed, and it is provided in Table 10.

(3) Knowledge transfer

**Table 10:** Knowledge storage measurement scale.

Variables	Label	Definition
Knowledge storage	CC1	Better knowledge storage systems (electronic, textual) within our learning communities
	CC2	I can learn what I need to know quickly through group e-learning.
	CC3	When I need to know something, I can quickly think of other students who have that knowledge.

The process of knowledge transfer within the learning community involves the flow and distribution of knowledge. Knowledge transfer is instrumental in advancing learning within the group and elevating the collective knowledge level, as well as in the effective utilization of knowledge. To evaluate and measure these aspects, a Knowledge Transfer Measurement Scale has been devised, and it is detailed in Table 11.

**Table 11:** Knowledge transfer measurement scale.

Variables	Label	Definition
knowledge transfer	ZY1	Students with a large knowledge base will share their knowledge with other students
	ZY2	We often use electronic networks to discuss or seek knowledge and to help
	ZY3	After a phase of learning, we transfer and apply the accumulated knowledge to the next phase

##### 3.2.3.5 Intellectual silence

Intellectual silence possesses distinctive features, including situational dependence, lack of logical structure, non-public nature, and inability to be conveyed through standard explicit organization. This type of knowledge is more challenging for peers to locate and comprehend, and as a result, intellectual silence impacts the formation of TMS. Consequently, an Intellectual Silence Measurement Scale has been crafted and is provided in Table 12.

**Table 12:** Intellectual silence measurement scale.

Variables	Label	Definition
Intellectual silence	JM1	Certain knowledge needs to be comprehended and mastered in group discussions
	JM2	Specialized teacher instruction is required for certain knowledge acquisition

##### 3.2.3.6 Effectiveness of TMS

To gauge the effectiveness of the TMS, three critical dimensions, namely Specialization, Credibility, and Coordination, are taken into consideration. A measurement scale has been devised to evaluate the TMS's validity, as detailed in Table 13.

**Table 13:** TMS effectiveness measurement scale.

Variables	Label	Definition
Effectiveness of TMS	YL1	Team members have specialized areas of knowledge in which they excel
	YL2	I have a great deal of trust in the knowledge possessed by other students in my learning community
	YL3	Our learning community can coordinate well and complete learning tasks efficiently

## 4 Empirical analysis

### 4.1 Data collection

The questionnaire used in this study was primarily an electronic survey tool for data collection. Students who had participated in online asynchronous learning completed the questionnaire based on their prior experiences with online asynchronous learning. The questionnaire consisted of two key sections: the first was "Basic Information", and the next was the "Scale Survey".

The Scale Survey was designed using a five-point Likert scale. Each question in the questionnaire was linked to the specific variable measurement indices outlined in Section 3. Respondents provided their answers on a five-point scale, ranging from "very non-compliant" to "very compliant." Furthermore, the questionnaire design in this study aimed to uphold the principles of selecting appropriate indicator questions and crafting clear, easily comprehensible questions.

This study selects the survey location of Northeast China and obtains data by distributing questionnaires to undergraduate, master's, and doctoral students. During the epidemic of COVID-19, the respondents' learning time and place broke through the traditional classroom limitations, experienced online asynchronous learning, and fully utilized the interactive memory mode to acquire knowledge. Therefore, the selection of this population is credible. Out of a total of 280 questionnaires distributed, 264 questionnaires were collected. After filtering out some incomplete and excessively similar responses, 229 questionnaires were deemed as effectively answered. This represents 82 % of all the distributed questionnaires.

### 4.2 Data analysis

SPSS can easily handle large-scale datasets, including data import, data cleaning, variable management, and other functions, which helps to improve data accuracy [41]. Its principle is to assume that A has no effect on B [42], if the analysis yields a result of P (sig) < 0.001/0.01/0.05, the hypothesis is not valid, i.e., A has a significant effect on B. If sig. = 0.531 is greater than >0.05, it means that the hypothesis is true that A has no effect on B (or B on A) and that changes in either party do not affect the other. It is in line with the relevant hypothesis judgment needs of this study.

Structural equation modeling (SEM) is a method for building, estimating, and testing causal models, which consists of a measurement and structural model [43]. The measurement model is used to describe the relationships between the latent variables and their corresponding observed indicators. In addition, the structural model is used to represent the relationships between latent variables. SEM can replace multiple regression, through-trail analysis, factor analysis, analysis of covariance and other methods to clearly analyze the role of individual indicators on the overall and the interrelationships between individual indicators.

The sample data in this study encompasses the results of the survey statistics related to the 33 measures corresponding to the 12 variables outlined in the hypothetical model. For data analysis, SPSS 27.0 software was employed to examine the basic characteristics, credibility, and validity of the data. Additionally, Amos 27.0 software [44] was used for structural equation model (SEM) analysis, including evaluating the model fit, assessing the coefficients of the model paths, and validating the hypotheses.

#### 4.2.1 Sample descriptive statistics

The questionnaire was administered to a cohort of students with experience with online asynchronous learning. As shown in Table 14, this group comprised 163 undergraduate students and below, 52 master's degree students, and 14 doctoral students. The gender distribution was nearly equal, with a balanced male-to-female ratio. The participants in the study were generally in the age range of 18–27 years old.

**Table 14:** Participant Demographics.

Feature	Categories	Numbers	Percentage
Gender	Male	113	49.34 %
	Female	116	50.66 %
Age	<25 years	184	80.35 %
	25–30 years	33	14.41 %
	>30 years	12	5.24 %
Level of education	Undergraduate and below	163	71.18 %
	Master's degree	52	22.71 %
	Doctor's degree	14	6.11 %

The results of the sample descriptive statistics are presented in Table 15. The mean, standard deviation, and variance values corresponding to the 33 measures are relatively small, and the values for each measure are close to each other. This is a consequence of the questionnaire design in this dissertation, which employed a Likert five-level scale. The data associated with various indicators exhibit small differences, resulting in low dispersion. The skewness values in the table are all less than 0, and some have a relatively large absolute value. This indicates that the distribution of sample data is skewed and has a negative skewness, suggesting an overall asymmetry. Most of the kurtosis values are less than 0, indicating that the distribution of the sample data is flatter than the peak of a normal distribution. This is influenced by the relatively high degree of similarity among the questionnaire respondents. In summary, the data does not follow a normal distribution pattern.

**Table 15:** Sample descriptive statistics.

Measurement indicators	N	Mean	Std dev	Var	Skewness	Kurtosis
QT1	229	3.62	. 960	0.972	−0.442	−0.486
QT2	229	3.82	0.956	0.914	−0.598	0.279
QT3	229	3.58	0.939	0.979	−0.289	−0.535
GT1	229	3.74	0.964	0.929	−0.501	−0.028
GT2	229	3.72	0.970	0.941	−0.364	−0.321
GT3	229	3.65	0.987	0.974	−0.357	−0.421
XR1	229	3.87	0.882	0.778	−0.446	−0.116
XR2	229	3.90	0.860	0.740	−0.514	0.309
XR3	229	3.68	0.982	0.964	−0.474	−0.183
NJ1	229	3.70	0.948	0.797	−0.618	0.053
NJ2	229	3.72	0.994	0.750	−0.599	0.076
NJ3	229	3.95	0.880	0.774	−0.491	−0.123
CB1	229	3.86	0.917	0.840	−0.546	0.025
CB2	229	3.80	0.918	0.843	−0.492	0.108
CB3	229	3.82	0.894	0.800	−0.559	0.360
GX1	229	3.89	0.951	0.905	−0.767	0.443
GX2	229	4.07	0.848	0.719	−0.648	0.233
HY1	229	4.01	0.845	0.715	−0.640	0.340
HY2	229	3.87	0.892	0.795	−0.347	−0.339
CC1	229	3.94	0.876	0.768	−0.590	−0.120
CC2	229	3.82	0.878	0.770	−0.467	−0.161
CC3	229	3.79	0.944	0.892	−0.493	−0.186
JM1	229	3.89	0.918	0.843	−0.536	−0.024
JM2	229	4.09	0.841	0.706	−0.756	0.534
CZ1	229	3.96	0.826	0.682	−0.484	0.205
CZ2	229	3.94	0.846	0.716	−0.541	0.216
CZ3	229	3.89	0.904	0.817	−0.573	0.130
ZY1	229	3.87	0.906	0.822	−0.460	−0.067
ZY2	229	4.14	0.833	0.694	−0.735	0.387
ZY3	229	3.99	0.830	0.688	−0.487	0.129
YL1	229	3.91	0.861	0.742	−0.570	0.401
YL2	229	3.87	0.902	0.813	−0.508	0.044
YL3	229	3.90	0.882	0.778	−0.412	−0.027

#### 4.2.2 Reliability and validity analysis

(1) Reliability Analysis

To evaluate the consistency, stability, and reliability of the sample data, SPSS 27.0 was employed. The reliability test was conducted using Cronbach's alpha coefficient, which was computed as shown in Equation (1).

(1) $${Cronbach}^{\prime }s\;\alpha =\frac{k}{k-1}\left(1-\frac{\sum_{i=1}^{k}{S_{i}}^{2}}{{S_{x}}^{2}}\right)=\frac{k}{k-1}\left(1-\frac{\sum_{i=1}^{k}{\delta_{i}}^{2}}{\sum_{i=1}^{k}{\delta_{i}}^{2}+2\sum_{i}^{k}\sum_{j}^{k}\delta_{ij}}\right)$$

Cronbach's α is a statistic used to gauge the internal consistency of a scale or test, providing insights into the data's reliability. Cronbach's α values range from 0 to 1. A value greater than 0.7 is generally indicative of good reliability. Values within the range of 0.35–0.7 suggest fair reliability, whereas values below 0.35 are often considered to represent poor reliability.

The reliability test of the research variables in this study is presented in Table 16. The table indicates that Cronbach's α value for each variable and its corresponding measures is above 0.7, signifying good reliability. Additionally, the Cronbach's α values after deleting individual items are lower than the overall Cronbach's α, reinforcing the conclusion that the overall reliability of the variables is satisfactory.

(2) Validity Analysis

**Table 16:** Table of reliability tests for research variables.

Variables	ZLable	Cronbach's α	After deleting Cronbach's α	Variables	Lable	Cronbach's α	After deleting Cronbach's α
Group learning		0.855		Knowledge storage		0.879	
	QT1		0.833		CC1		0.869
	QT2		0.740		CC2		0.822
	QT3		0.819		CC3		0.790
Group communication		0.873		Knowledge creation		0.861	
	GT1		0.813		CZ1		0.788
	GT2		0.758		CZ2		0.783
	GT3		0.780		CZ3		0.844
Membership trust		0.853		Knowledge transfer		0.850	
	XR1		0.751		ZY1		0.797
	XR2		0.772		ZY2		0.836
	XR3		0.852		ZY3		0.734
Group cohesion		0.872		Task interdependence		0.869	
	NJ1		0.780		HY1		
	NJ2		0.723		HY2		
	NJ3		0.820				
Shared Willingness		0.769		Intellectual silence		0.765	
	GX1				JM1		
	GX2				JM2		
Knowledge stock		0.909		Effectiveness of TMS		0.899	
	CB1		0.869		YL1		0.868
	CB2		0.839		YL2		0.857
	CB3		0.899		YL3		0.844

Note: "Label" represents the measurement indicators of each variable and serves as the abbreviation for the evaluation dimension of the measurement scale described in Section 3.2.3.

Validity analysis was conducted using SPSS 27.0 software to determine whether the measures can accurately represent and explain the variables and the extent to which they can provide explanatory power. Two commonly used tests for validity analysis are the Kaiser-Meyer-Olkin (KMO) test and Bartlett's test for sphericity.

KMO Test: The KMO (Kaiser-Meyer-Olkin) value evaluates the degree of validity. A KMO value exceeding 0.8 suggests a high level of validity, while a value in the range of 0.6–0.7 indicates a reasonable level of validity. A KMO value below 0.6 is indicative of poor validity.

Bartlett's Test of Sphericity: When Bartlett's test of sphericity is significant (at the 0.05 level), it rejects the null hypothesis, signifying that there is a correlation between the variables that are conducive for factor analysis.

The outcomes of the KMO test and Bartlett's sphericity test can be found in Table 17, Table 18, respectively.

**Table 17:** KMO test and Bartlett's test of sphericity for research variables.

Variables	KMO value	Bartlett's Sphericity Test	Bartlett Sphericity Test	Bartlett Sphericity Test
		χ^2^	df	Sig
Group learning	0.709	322.430	3	<0.001
Group communication	0.692	402.181	3	<0.001
Membership trust	0.712	323.291	3	<0.001
Group cohesion	0.668	416.642	3	<0.001
Knowledge stock	0.743	466.218	3	<0.001
Knowledge creation	0.728	322.992	3	<0.001
Knowledge storage	0.728	370.360	3	<0.001
Knowledge transfer	0.710	305.937	3	<0.001
Effectiveness of TMS	0.752	419.350	3	<0.001

**Table 18:** Sample overall KMO test and Bartlett's sphericity test.

KMO value		0.960
Bartlett Sphericity Test	χ^2^	7411.503
	Df (degree of freedom)	528
	Sig (significance probability)	0.000

As shown in Table 17, the KMO test values for the study variables are all above 0.6, indicating that the validity of the variables is acceptable. However, for the three variables - willingness to share, task interdependence, and Intellectual silence - it's not appropriate to test their validity as they have only two observables.

Table 18 indicates that the KMO test value is 0.960, exceeding 0.8. This high value suggests that the sample data exhibits a high level of validity. Furthermore, Bartlett's test of sphericity yields a significance probability of 0.000, leading to the rejection of the null hypothesis at the 0.05 level. The test result suggests a meaningful relationship between the variables, making them suitable for factor analysis. In summary, the comprehensive analysis shows that the overall validity of the sample data is good.

### 4.3 Model fitting and hypothesis validation

Structural Equation Modeling (SEM) is a powerful statistical technique that amalgamates two primary analytical approaches: factor analysis and path analysis. SEM enables the investigation of relationships between variables and the evaluation of how accurately a proposed model aligns with the observed data. In this study, Amos 27.0 software is employed to analyze various aspects of the hypothetical model related to the online asynchronous learning TMS. This analysis includes evaluating the model fit, hypothesis testing, and conducting path analysis to examine the relationships between different variables. SEM provides a comprehensive approach to understanding and testing complex models, making it a valuable tool in research and analysis.

#### 4.3.1 Analysis of model fitting results

The evaluation of a structural equation model's fit can be conducted in two main ways.

(1) Testing Relevant Parameter Estimates: In this approach, parameter estimates are tested to assess their significance. When most of the parameter values are found to be significant, it indicates that there are meaningful relationships between the variables, the model has a high degree of fit, and the conceptual model is considered reasonable. If any parameter values are not significant, it suggests that the model may need to be modified.
(2) Verifying Relevant Fit Measures: In this approach, various fit measures are used to assess how well the model aligns with the observed data. When these measures fall within a reasonable range based on predefined criteria, it indicates that the model has a high degree of fit. If the fit measures are outside the acceptable range, it suggests that the model may require modifications.

The criteria for assessing the model's goodness of fit can be found in Table 19. These criteria are important for assessing the overall quality of the model and determining whether adjustments are needed.

**Table 19:** Model fit evaluation.

Goodness-of-fit metrics	The goodness of fit evaluation
χ^2^	P > 0.05, Good fit
χ^2^/*df*	(1.0,3.0), Good fit
RMR	RMR<0.05, Good fit
RMSEA	(0.05,0.08), Fair fit; RMSEA<0.05, Good fit
GFI	GFI>0.9, Good fit
IFI or NFI	RFI or NFI >0.9, Good fit

The original structural equation model was initially analyzed using Amos 27.0 software, resulting in a low model fit. To address this issue, Amos software automatically identified and rejected abnormal Modification Indices (M.I.) values. These are typically the largest M.I. values that significantly exceed other similar values. The software then reruns the analysis after removing these problematic values. This process is repeated until the change in the model's fit becomes less significant. Furthermore, restricted, or fixed parameters were replaced with free parameter estimates, and the model's fit was repeatedly assessed. The corrected standardized regression coefficients are presented in Table 20.

**Table 20:** Table of standardized regression coefficients and significance P for models.

Relationships between the effects of variables	Standardized regression coefficients	P
Group learning --- > Knowledge creation	0.37	***
Group learning --- > Knowledge transfer	0.26	**
Group communication --- > Knowledge creation	0.55	***
Group communication --- > Knowledge transfer	0.23	**
Membership trust --- > Knowledge storage	0.60	***
Membership trust --- > Knowledge transfer	0.72	***
Group cohesion --- > Knowledge storage	0.55	***
Group cohesion --- > Knowledge transfer	0.04	0.03
Knowledge stock --- > Knowledge creation	0.25	**
Shared Willingness --- > Knowledge transfer	0.28	**
Intellectual silence --- > Effectiveness of TMS	−0.21	**
Task interdependence --- > Effectiveness of TMS	0.06	0.03
Knowledge storage --- > Effectiveness of TMS	0.04	0.02
Knowledge creation --- > Effectiveness of TMS	0.26	**
Knowledge transfer --- > Effectiveness of TMS	0.63	***

In Table 20, the path coefficients between the variables are presented as standardized regression coefficients. The significance of these coefficients is indicated by the associated p-values. Specifically.

(1) If the p-value corresponds to "***," which means that the path coefficient shows significance at the 0.001 threshold.
(2) If the p-value corresponds to "**," which means that the path coefficient shows significance at the 0.01 threshold.
(3) If the p-value corresponds to a specific value, it suggests that the path coefficient is not statistically significant at the 0.01 level.

In this study, a significance level of 0.01 is set. When the p-value corresponds to " ***" or "**," it suggests a strong and significant relationship between the variables [41].

As shown in Table 20, the model indicates that the relationships between group cohesion and knowledge transfer, task interdependence and the effectiveness of the TMS, and knowledge storage and the effectiveness of TMS are non-significant. However, the remaining variables in the model exhibit more significant and influential relationships with each other.

The model fit evaluation results are provided in Table 21. These steps were taken to refine the model and improve its overall fit to the observed data.

**Table 21:** Summary of model fit evaluation.

Indicators	*df*	χ^2^	P	χ^2^/*df*	RMR	GFI	RMSEA	NFI	IF	PGFI
Value	480	3020	0.000	6.2	0.000	0.931	0.052	0.912	0.834	0.407
Fitness			Poor	Poor	Good	Good	Acceptable	Good	Acceptable	Poor

As indicated in Table 21, the selected model fit indicators reveal that only three of them suggest that the model fit is not good, while the other five indicators indicate that the model fit is good or acceptable. Therefore, the overall fit of the model in this study can be considered as good. The less favorable fit results may, in part, be attributed to limitations in the survey data. Ensuring the objectivity of respondents when completing questionnaires can be challenging, and the data did not exhibit a perfect state of normal distribution. In conclusion, this study finds that the hypothesized model has a reasonably good fit, and the variables and their relationships within the model can be interpreted effectively.

#### 4.3.2 Analysis of hypothesis testing results

Table 22 provides an overview of the results obtained from hypothesis testing, and the hypothetical model path for the formation of an online asynchronous learning TMS is illustrated in Fig. 3.

**Table 22:** Analysis of results corresponding to hypothesis testing.

Hypothesis	Hypothetical content	Results
H1	Task interdependence is related to the effectiveness of TMS	Not satisfied
H2a	Knowledge creation is positively related to the effectiveness of TMS	Satisfied
H2b	Knowledge storage is related to the effectiveness of TMS	Not satisfied
H2c	Knowledge transfer is positively correlated with the effectiveness of TMS	Satisfied
H3	Intellectual silence is negatively correlated with the effectiveness of TMS	Satisfied
H4a	Group learning promotes knowledge creation and ultimately positively affects the effectiveness of TMS	Satisfied
H4b	Group learning promotes knowledge transfer and ultimately positively affects the effectiveness of TMS	Satisfied
H4c	Group communication promotes knowledge creation and ultimately positively affects the effectiveness of TMS	Satisfied
H4d	Group communication promotes knowledge transfer and ultimately positively affects the effectiveness of TMS	Satisfied
H4e	Membership trust promotes knowledge storage and ultimately positively affects the effectiveness of TMS	Satisfied
H4f	Membership trust promotes knowledge transfer and ultimately positively affects the effectiveness of TMS	Satisfied
H4g	Group cohesion promotes knowledge storage and ultimately positively influences the effectiveness of TMS	Satisfied
H4h	Group cohesion promotes knowledge transfer and ultimately positively affects the effectiveness of TMS	Not satisfied
H5a	Knowledge stock promotes knowledge creation and ultimately has a positive impact on the effectiveness of TMS	Satisfied
H5b	Shared Willingness promotes knowledge transfer and ultimately positively affects the effectiveness of TMS	Satisfied

**Fig. 3:** Plot of path coefficients for structural equations.

Table 20 provides an examination of the results from the hypothesis tests. The stronger the causal relationship between the variables, the closer the absolute value of the standardized regression coefficients gets to 1. Fig. 3 shows the standardized coefficients for each hypothetical path.

H1 The p-value for the impact of task interdependence on the effectiveness of the TMS is 0.03, which is not significant at the 0.01 level. Therefore, the original hypothesis, suggesting a significant relationship between task interdependence and the TMS, is not valid.

H2a The path coefficient representing the influence of knowledge creation on the effectiveness of the TMS is 0.26, signifying its significance at the 0.01 level. Hence, the original hypothesis is confirmed, suggesting a positive relationship between knowledge creation and the effectiveness of the TMS.

H2b The p-value for the impact of knowledge storage on the effectiveness of the TMS is 0.02, which is not significant at the 0.01 level. Thus, the original hypothesis, which proposed a significant relationship between knowledge storage and the TMS, is not valid.

H2c The path coefficient reflecting the effect of knowledge transfer on the effectiveness of the TMS is 0.63, which shows significance at the 0.01 significance level Therefore, the original hypothesis is confirmed, indicating a positive relationship between knowledge transfer and the effectiveness of the TMS.

H3 The path coefficient representing the impact of the degree of intellectual silence on the effectiveness of the TMS is −0.21, which shows significance at the 0.01 significance level. Consequently, the original hypothesis is validated, revealing a negative relationship between intellectual silence and the effectiveness of the TMS.

H4a The path coefficient for the influence of group learning on knowledge creation is 0.37, signifying its significance at the 0.01 level. Thus, the original hypothesis is confirmed, suggesting that group learning promotes knowledge creation and ultimately has a positive effect on the effectiveness of the TMS.

H4b The path coefficient reflecting the impact of group learning on knowledge transfer is 0.26, signifying its significance at the 0.01 level. Therefore, the original hypothesis is confirmed, indicating that group learning facilitates knowledge transfer and ultimately has a positive effect on the effectiveness of the TMS.

H4c The path coefficient representing the influence of group communication on knowledge creation is 0.55, signifying its significance at the 0.01 level. Thus, the original hypothesis is confirmed, revealing that group communication promotes knowledge creation and ultimately has a positive effect on the effectiveness of the TMS.

H4d The path coefficient indicating the effect of group communication on knowledge transfer is 0.23, signifying its significance at the 0.01 level. Hence, the original hypothesis is confirmed, showing that group communication facilitates knowledge transfer and ultimately has a positive effect on the effectiveness of the TMS.

H4e The path coefficient reflecting the impact of member trust on knowledge storage is 0.60, signifying its significance at the 0.01 level. Therefore, the original hypothesis is confirmed, indicating that member trust promotes knowledge storage and ultimately has a positive effect on the effectiveness of the TMS.

H4f The path coefficient representing the influence of member trust on knowledge transfer is 0.72, which shows significance at the 0.01 significance level Consequently, the original hypothesis is confirmed, revealing that member trust facilitates knowledge transfer and ultimately has a positive effect on the effectiveness of the TMS.

H4g The path coefficient indicating the effect of group cohesion on knowledge storage is 0.55, signifying its significance at the 0.01 level. Thus, the original hypothesis is confirmed, suggesting that group cohesion promotes knowledge storage and ultimately has a positive effect on the effectiveness of the TMS.

H4h The p-value of the path coefficient representing the impact of group cohesion on knowledge transfer is 0.03, which is not significant at the 0.01 level. Therefore, the original hypothesis, which proposed a significant relationship between group cohesion and knowledge transfer, is not valid.

H5a The path coefficient reflecting the influence of the knowledge stock on knowledge creation is 0.25, signifying its significance at the 0.01 level. Hence, the original hypothesis is confirmed, revealing that knowledge stockpile promotes knowledge creation and ultimately has a positive effect on the effectiveness of the TMS.

H5b The path coefficient indicating the effect of willingness to share on knowledge transfer is 0.28, which shows significance at the 0.01 significance level Consequently, the original hypothesis is confirmed, indicating that willingness to share facilitates knowledge transfer and ultimately has a positive effect on the effectiveness of TMS.

## 5 Discussion

Based on the analysis of the path coefficients presented in Fig. 3, we can conclude that group learning, group communication, membership trust, and group cohesion significantly influence knowledge creation, storage, and transfer to a certain degree. These factors contribute to enhancing the knowledge management capabilities of the learning group and ultimately positively impact the effectiveness of the TMS.

(1) Analysis of findings

The result shows that H1, H2a, H2c, H3, H4a, H4b, H4c, H4d, H4f, H4g, H5a, H5b support the original hypothesis, but H2a, H4b, H4d, H5a, H5b correlation coefficients are low (less than 0.3), which may be due to the fact that the study was investigated as a result of a specific single online learning context, which was influenced by the limitations of the context of use, making the correlation coefficients low. However, hypotheses H1, H2b, and H4h are not satisfied, which could be due to the following reasons.

H1 There is no significant relationship between task interdependence and TMS effectiveness, which may be due to the significant differences in cognitive abilities and knowledge levels among team members [45], making it difficult for TMS to work effectively.

H2b Even if the team has a well-developed knowledge storage system, the effectiveness of the TMS will still be compromised if members are not willing to share knowledge or actively use that stored knowledge [46]. The effectiveness of the TMS relies on active interaction and collaboration among members, not just the storage of knowledge.

H4h In cohesive teams, members may be too dependent on others and lack autonomy and initiative [47]. This dependence can lead to less efficient information transfer and knowledge sharing.

(2) The impacts of group factors on the development of online asynchronous learning TMS

The findings suggest that group factors positively influence the effectiveness of interactive memory systems. Group learning primarily involves the process of knowledge creation, contributing positively to the collective expertise within the TMS, and enhances communication among members, deepening their mutual understanding and, subsequently, facilitating knowledge transfer and improving group coordination. Group communication serves as a pivotal factor for knowledge transfer, allowing learning members to make the most of their knowledge by effectively interacting with one another. Active and efficient communication among learning members is crucial for fostering the TMS in online asynchronous learning, which often involves numerous diverse individuals.

Effective knowledge exchange among group members is contingent upon trust in the knowledge held by fellow members. Membership trust stands as a prerequisite for successful team knowledge transfer, with a higher degree of membership trust further facilitating the formation of the TMS. Additionally, group cohesion, reflecting the overall learning atmosphere and the degree of cohesion among members, significantly impacts the coordination of the TMS. A strong sense of group cohesion promotes the development of the TMS in online asynchronous learning.

(3) The impacts of individual factors and knowledge management on the development of online asynchronous learning TMS

Individual factors, specifically knowledge stock and shared willingness, correlate positively with the effectiveness of TMS. The level of expertise that individuals bring to the learning environment significantly contributes to the achievement of learning objectives. The cumulative sum of individual knowledge stocks forms an integral part of the overall knowledge base within the group, reflecting the diverse expertise present in the TMS.

The shared willingness of individuals plays a pivotal role in facilitating knowledge transfer among group members. A strong shared willingness is a powerful motivator for learning members to exchange knowledge with their peers, thereby fostering the formation of a robust TMS.

(4) The Impacts of intellectual silence on the development of online asynchronous learning TMS

A positive correlation exists between the degree of intellectual silence and the establishment of TMS. In certain scenarios, the level of intellectual silence can directly influence the creation and effectiveness of TMS. When the degree of intellectual silence is low, meaning that individuals or organizations are more inclined to share their knowledge and experiences, the formation of TMS progresses more seamlessly. This is because knowledge sharing facilitates the flow and dissemination of information, thereby providing additional content and resources for the development of TMS. Consequently, the TMS becomes richer and more valuable.

(5) The impacts of task interdependence on the development of online asynchronous learning TMS

The relationship between task interdependence and the formation of TMS exhibits a degree of incongruity. TMS are typically designed to facilitate knowledge sharing, collaboration, and cross-domain learning and are not strictly contingent on task-specific interdependencies. The principal aim of TMS is to enable the accumulation, transfer, and sharing of knowledge within the framework of a learning community or organization. This process primarily hinges on the willingness and culture of the individual or organization, as well as the support of a technological platform, rather than being predicated solely on interdependencies between specific tasks. Consequently, task interdependencies do not directly influence the formation and efficient operation of the TMS. Instead, establishing a positive culture of knowledge sharing, which encourages individuals and organizations to disseminate their knowledge and experiences, is paramount in promoting system development and enhancing knowledge management effectiveness. While task interdependence may play a role, it is not the sole determinant.

(6) The impacts of knowledge management on the development of online asynchronous learning TMS

The results indicate that knowledge management, as a mediating variable, has a significant impact on the effectiveness of interactive memory systems, which can enhance the learning and memory effects of interactive memory systems and improve the overall learning experience and effectiveness by facilitating knowledge creation, optimizing knowledge storage, and facilitating knowledge transfer.

Knowledge creation through teamwork and innovative thinking can provide richer and more diverse learning resources for interactive memory systems [48]. Knowledge storage [49] allows interactive memory systems to access and utilize existing knowledge resources more efficiently, which helps to improve learning and memorization effects. Knowledge is transferred from one environment or individual to another, and is disseminated and shared in an interactive memory system, thus enhancing communication and interaction between learners, and improving learning efficiency [50].

(7) Limitations and future work

The factors influencing the hypothetical model of the TMS have been derived from a synthesis of existing literature on TMS, knowledge management, and online asynchronous learning. However, additional factors, such as member psychology, study habits, and teaching strategies, may also impact the formation of the TMS in the context of online asynchronous learning [51]. Moreover, SPSS analysis is often inadequate for handling large-scale and complex data, while SEM analysis may be less accurate for small-sample data, potentially affecting the accuracy of the results. Future research could expand the model to include a broader spectrum of influencing factors, integrating multiple disciplines such as psychology and computer science to explore the TMS further. This approach could advance the development and application of online education and learning technologies.

## 6 Conclusion

This study meticulously organized and analyzed existing research on TMS, while synthesizing pertinent knowledge management theories. The primary aim was to pinpoint the fundamental factors influencing the establishment of TMS within the realm of online asynchronous learning. To achieve this, the study harnessed SPSS data analysis and structural equation modeling, conducting a comprehensive empirical analysis to reveal the real-world impact of each influencing factor on the formation of TMS. As a result, a series of significant findings regarding the formation of TMS in online asynchronous learning emerged. These key results include.

(1) The adaptation of TMS to the realm of online asynchronous learning, coupled with their integration with knowledge management principles to unravel the formation process of TMS in this specific context, with knowledge management acting as a mediating variable.
(2) Following the research framework of "group factors - individual factors - knowledge management - task interdependence - intellectual silence - effectiveness of TMS," the study successfully constructed a conceptual model and a hypothetical model for the formation of TMS in online asynchronous learning. Furthermore, it effectively identified the pivotal factors influencing the establishment of these systems.

This study serves as a critical cornerstone for gaining a more profound understanding of online asynchronous learning environments. By elucidating the factors that impact the development and operation of TMS, educators can enhance the customization of course designs and the allocation of learning resources. Such personalization can cater to the diverse needs and learning preferences of students, ultimately leading to improved educational outcomes. Additionally, these findings offer valuable insights for educational policymakers, enabling them to discern the factors that influence learning outcomes and experiences in the realm of online asynchronous learning. Armed with this knowledge, policymakers can develop targeted strategies and measures to better cater to learners' needs and enhance their overall learning experience. This, in turn, can drive ongoing enhancements and innovations in the sphere of online education.

## Ethics statement

This study was reviewed and approved by the ethics committee of School of Maritime Economics and Management, Dalian Maritime University, with the approval number: [2023001].

## Data availability statement

All the relevant data are included in the manuscript and the supplementary document. No separate repository is attached.

## CRediT authorship contribution statement

**Jiao Zhang:** Writing – original draft, Software, Methodology, Investigation, Funding acquisition, Formal analysis, Data curation, Conceptualization. **Min Zhao:** Writing – review & editing, Supervision, Funding acquisition. **Liang Wang:** Writing – review & editing, Supervision, Funding acquisition, Conceptualization.

## Declaration of competing interest

The authors declare that they have no known competing financial interests or personal relationships that could have appeared to influence the work reported in this paper.
